# Diagnostic Value of Peripheral Blood Lymphocytes for Primary Immune Thrombocytopenia

**DOI:** 10.1155/2022/9833941

**Published:** 2022-08-16

**Authors:** Jun Lu, Ling Sun, Xifeng Wu, Tantan Li, Lijie Men

**Affiliations:** ^1^Jinan People's Hospital Affiliated to Shandong First Medical University, Jinan, China; ^2^Jinan City People's Hospital, Jinan, China

## Abstract

The purpose of this study was to investigate the absolute value of peripheral blood lymphocytes in patients with primary immune thrombocytopenia and the diagnostic effect on patients with primary immune thrombocytopenia. From January 2020 to June 2021, 76 patients with primary immune thrombocytopenia and 80 healthy check-ups admitted to our hospital were selected as study subjects and divided into a control group (80 patients, healthy check-ups) and an observation group (76 patients, primary immune thrombocytopenia), according to the health status of the organism. Early morning fasting venous blood was collected from both groups, and the absolute value of peripheral blood lymphocytes was measured and compared using a fully automated hematology analyzer to investigate the diagnostic value of absolute peripheral blood lymphocytes in primary immune thrombocytopenia. The CD3+, CD3+CD4+, CD4+/CD8+, and CD16+CD56+ assay values in the observation group were lower than those in the control group, and the CD3+CD8+, CD19+, and ALC assay values were higher than those in the control group (*P* < 0.05). The CD3+CD8+ detection values of newly diagnosed patients were similar to those of relapsed refractory patients (*P* > 0.05); CD3+, CD3+CD4+, CD4+/CD8+, and CD16+CD56+ detection values of newly diagnosed patients were lower than those of relapsed refractory patients, and CD19+ and ALC detection values were higher than those of relapsed refractory patients; CD3+, CD3+CD4+, CD4+, CD4+/CD8+, and CD16+CD56+ detection values of mild patients were lower than those of relapsed refractory patients; CD3+, CD3+CD4+, CD4+/CD8+, and CD16+CD56+ detection values were higher in mild patients than in severe patients, and CD3+CD8+, CD19+, and ALC detection values were lower than in severe patients (*P* < 0.05). The absolute lymphocyte values were of high diagnostic value in primary immune thrombocytopenia, with a sensitivity and specificity of 93.42% and 90.00%. The application of absolute peripheral blood lymphocyte value in the clinical diagnosis of primary immune thrombocytopenia can achieve a better detection and diagnosis effect, which has a positive impact on the early diagnosis rate and can help patients to obtain more timely, effective and targeted treatment, and is worthy of promotion.

## 1. Introduction

Primary immune thrombocytopenia is a common bleeding disorder caused by reduced platelet counts, with typical clinical manifestations of generalized bleeding from multiple mucosal skin sites and weakness. If not treated promptly, the disease can lead to organ bleeding or even intracranial hemorrhage as it worsens, posing a serious threat to patients' lives [1, 2]. As research has progressed, it has been found that primary immune thrombocytopenia is closely related to infections, immune responses to platelet-associated antigens and platelet-reactive T cells [3, 4]. Absolute peripheral blood lymphocyte values can effectively reflect the levels of T and B lymphocytes and can help physicians to assess the immune function of the subject [5, 6]. The application of absolute peripheral blood lymphocyte values to primary immune thrombocytopenia can help physicians to assess and diagnose the immune mechanism of the subject, there are few studies on absolute peripheral blood lymphocyte values in primary immune thrombocytopenia, but they have a small number of patients and are mostly the result of a few studies abroad, with very little research on this in China. Therefore, in this study, we propose to investigate the diagnostic value of absolute peripheral blood lymphocyte values in this condition by comparing 76 patients with primary immune thrombocytopenia admitted to our hospital from January 2020 to June 2021 and 80 healthy subjects.

## 2. Patients and Methods

### 2.1. Patients

From January 2020 to June 2021, 76 patients with primary immune thrombocytopenia and 80 healthy check-ups admitted to our hospital were selected as study subjects. Patients met the diagnostic criteria for primary immune thrombocytopenia in “Research and diagnosis of primary immune thrombocytopenia: an international consensus report” [7], including routine blood tests showing ≥2 decreases in platelet count and no abnormal blood cell morphology, generally no enlargement of the spleen, and bone marrow tests suggesting an increased or normal megakaryocyte count and impaired maturation. Inclusion criteria were as follows: (i) patients were aged 18–70 years; (ii) patients had typical symptoms such as bleeding from multiple parts of the mucous membranes and skin throughout the body; (iii) basic information was complete; (iv) study subjects and family members voluntarily signed an informed notice. Exclusion criteria were as follows: (1) patients were diagnosed with other secondary thrombocytopenia, such as proliferative diseases of the lymphatic system and malignant hematological diseases; (2) patients received medical treatment affecting the immune mechanism of the organism within 1 month before this study; (3) patients had a history of severe allergies, or suffered from autoimmune diseases such as allergic rhinitis; (4) patients had psychiatric disorders and too poor compliance. According to the health status of the organism, the group was divided into a control group (80 cases, healthy physical examiners) and an observation group (76 cases, primary immune thrombocytopenia). The differences were not statistically significant (*P* > 0.05) when comparing the basic information of the two groups, such as age, body mass index, gender composition, and education level (Table 1). The study was approved by the medical ethics committee.

### 2.2. Method

The study subjects were all subjected to absolute peripheral blood lymphocyte testing, which was performed as follows: (1) Apparatus and reagents: low-speed centrifuge (Beckman Coulter, model Microfuge 20/20R); fully automatic hematology analyzer (Myriad, model BS-280); spiral shaker (Jiangyan Xinkang Medical Equipment Co. Ltd., model TW3); hemolysin (BD FACSTM Lysing Solution); monoclonal six-colour antibody (BD Multisets TM 6-color TBNK Ragent); absolute counting tubes (BD TrucountTM Tubes); micro pipette (VTTLAB, Germany, 20/200/1000 *μ*L). (2) Assay method: peripheral venous blood was collected early in the morning on a fasting basis (≥6 h fasting) and placed in anticoagulated tubes, 2 ml/tube, 2 tubes in total. The blood sample (50 *μ*L) was added to the absolute count tube using a micropipette, 10 *μ*L of monoclonal hexachromatic antibody was added and mixed on a spiral shaker, protected from light for 15 min, at room temperature. Afterwards, 450 *μ*L of hemolysin was added, mixed, and kept away from light for 15 min at room temperature. Finally, the lymphocytes were tested using a low-speed centrifuge and a fully automated hematology analyzer.

### 2.3. Observation Indicators

The absolute values of lymphocytes in the two groups were compared: the levels of T lymphocytes (CD3+, CD3+CD4+, CD3+CD8 +, CD4+/CD8+), B lymphocytes and natural killer (NK) cells (CD19+, CD16+CD56 +), and the absolute value of lymphocytes (ALC) just after admission were statistically measured in the two groups.

The absolute lymphocyte counts of patients with different diseases in the observation group were compared: the CD3 +, CD3 + CD4 +, CD3 + CD8 +, CD4 +/CD8 +, CD19 +, CD16 + CD56 + and ALC levels of newly diagnosed (admission diagnosis of primary immune thrombocytopenia ≤1 year), relapsed and refractory (relapse after 5 years of follow-up after completion of diagnosis and treatment and discharge), mild (platelet count ≥30 × 10/L), and severe (platelet count <30 × 10/L) patients were counted. To analyze the diagnostic value of absolute value of peripheral blood lymphocytes in primary immune thrombocytopenia, the diagnostic results of platelet combined with bone marrow examination were regarded as the gold standard, the diagnostic value of absolute value of peripheral blood lymphocytes was compared, and the sensitivity, specificity, positive prediction, and negative prediction were calculated.

### 2.4. Statistical Analysis

Statistical Product and Service Solutions (SPSS) 23.0 (IBM, Armonk, NY, USA) was applied for statistical analysis. Independent sample *t*-test was used for comparison between groups for measurement data obeying normal distribution, and independent sample *t*-test was used for comparison within groups, all expressed as ($\bar{x}$ ± *s*). Count data were tested by *χ*^2^ and expressed as rate (%), and *P* < 0.05 indicates statistical difference.

## 3. Results

### 3.1. Lymphocytes in the Two Groups

The detection values of CD3+, CD3+ CD4+, CD4+/CD8+, and CD16+CD56+ in the observation group were lower than those in the control group, and the detection values of CD3+CD8+, CD19+, and ALC were higher than those in the control group, and the differences had statistical significance (*P* < 0.05) (Table 2).

### 3.2. Lymphocytes in Patients with Different Diseases in the Observation Group

The CD3+CD8+ detection values of newly diagnosed patients were similar to those of relapsed and refractory patients, and the difference was not statistically significant (*P* > 0.05). The detection values of CD3+, CD3+CD4+, CD4+/CD8+, and CD16+CD56+ in newly diagnosed patients were lower than those in relapsed and refractory patients, and the detection values of CD19+ and ALC were higher than those in relapsed and refractory patients; the detection values of CD3+, CD3+CD4 +, CD4+/CD8+, and CD16+CD56+ in mild patients were higher than those in severe patients, and the detection values of CD3+CD8+, CD19+, and ALC were lower than those in severe patients, and the differences were statistically significant (*P* < 0.05) (Tables 3 and 4).

### 3.3. The Diagnostic Value of Absolute Peripheral Blood Lymphocytes in Primary Immune Thrombocytopenia

The diagnostic value of absolute lymphocyte count in primary immune thrombocytopenia was high, with a sensitivity and specificity of 93.42% and 90.00% (Tables 5 and 6).

## 4. Discussion

Primary immune thrombocytopenia is an acquired autoimmune disease. In addition to the negative correlation between platelet autoantibodies and platelet counts, the incidence of primary immune thrombocytopenia is increased by platelet-reactive T cells, immune reactions to platelet-associated antigens that cause thrombocytopenia, and natural immune defenses caused by viral infections [8]. Patients with acute thrombocytopenia are more likely to have an acute onset and duration of illness of less than 6 months, and are more likely to become chronic if the disease remains untreated. As the disease worsens and the number of thrombocytopenia increases, the coagulation-anticoagulation balance in the patient's body is severely disrupted and the patient's life is seriously threatened.

In order to improve the early diagnosis of primary immune thrombocytopenia, this study proposed to apply the absolute peripheral blood lymphocyte values to the clinical diagnosis of this condition. In this study, a series of findings suggest that lymphocyte levels were closely associated with the development and progression of primary immune thrombocytopenia. This may be due to the fact that (1) lymphocytes are a type of leukocyte, produced mainly by lymphoid organs, are an important cellular component of the body's immune response function, and are the main performers of the immune function [9, 10]. In terms of physiology, but in the presence of pathogenic microorganisms, cancer cells, and allogeneic cells in the human body, lymphatic T cells and B cells were transformed and differentiated into allergenic T lymphocytes, plasma cells, and immunoglobulins to remove the invading substances, participate in humoral immunity and reduce the degree of damage to the organism, while NK cells have the role of killing target cells and are important in promoting the recovery of the inflammatory response and maintaining the health of the organism [11]. NK cells have a role in killing target cells and are important for the recovery of the inflammatory response and the maintenance of the body's health. Thus, in patients with primary immune thrombocytopenia, the number of lymphocyte subpopulations and the absolute value of lymphocytes may be abnormal when platelets are reduced as a result of immune reactions to viral infections and platelet-associated antigens. (2) Excessive immune-mediated destruction of platelets and decreased platelet counts by humoral and cellular abnormalities are important factors contributing to primary immune thrombocytopenia. CD3+, CD4+, CD8+, CD19+, CD16+, and CD56+ are common markers of lymphocytes, and testing for changes in the levels of these lymphocyte subsets can provide an important reference for the clinical diagnosis of the patient's immune function. CD3+ is a common marker of lymphocytes. Meanwhile, CD3+ can be involved in transmitting T cell activation signals and mediating various immune responses; CD4+ and CD8+ are closely related to inflammatory responses and hypersensitivity reactions, and decreasing levels of CD3+, CD3+CD4+, CD4+/CD8+, and increasing levels of CD3+CD8+ indicate an increase in platelet destruction mediated by CD8+ cytotoxic T cells and a significant decrease in platelet count [12]. CD16+ and CD56+ are involved in antitumor and anti-infection immune responses; CD19+ is associated with hyperactive liquid immunity, and an increase in CD19+ and a decrease in CD16+CD56+ levels indicates an increase in hyperactive liquid immunity, an abnormal expression of the body's immunity, a weakened antitumor and anti-infection immune response, and severe damage to the body [13, 14]. (3) The higher the ALC level, the more severe the primary immune thrombocytopenia. The higher the ALC level, the more severe the primary immune thrombocytopenia. This indicates that the ALC level can reflect the immune function of the subject and may provide an important reference for the clinical diagnosis of primary immune thrombocytopenia.

## 5. Conclusion

The application of absolute peripheral blood lymphocyte values to the clinical diagnosis of primary immune thrombocytopenia can achieve a more satisfactory detection and diagnosis effect, which has a positive impact on the early diagnosis rate and can help patients to obtain more timely, effective, and targeted treatment.

## Figures and Tables

**Table 1:** Comparison of basic data between the two groups (*x̅* ± *s*, *n*).

Group	Number of subjects	Age (years)		Body mass index (kg/m^2^)		Gender composition		Education level	
		Scope	Average	Scope	Average	Male	Female	≤College	≥Undergraduate
Observation group	76	18–67	42.56 ± 5.76	19–28	23.56 ± 1.86	41 (53.95%)	35 (46.05%)	48 (63.16%)	28 (36.84%)
Control group	80	20–70	44.93 ± 7.85	18–29	23.67 ± 1.97	47 (61.84%)	33 (43.42%)	45 (59.21%)	35 (46.05%)
Χ^2^*/t*	—	2.141		0.358		0.366		0.773	
*P* value	—	0.034		0.721		0.545		1.379	

**Table 2:** Comparison of the lymphocytes of the two groups (*x̅* ± *s*, cells/*μ*L).

Group	*n*	CD3+	CD3+CD4+	CD3+CD8+	CD4+/CD8+	CD19+	CD16+CD56+	ALC (×109/L)
Observation group	76	781.94 ± 115.89	485.78 ± 27.85	688.96 ± 32.75	1.06 ± 0.46	345.92 ± 37.84	245.87 ± 26.78	3.77 ± 0.82
Control group	80	1573.56 ± 152.43	689.83 ± 30.83	422.56 ± 27.04	1.86 ± 0.53	177.84 ± 27.47	403.01 ± 33.46	2.67 ± 0.54
*t*	—	36.374	43.305	55.517	10.046	31.864	32.280	9.943
*P* value	—	0.001	0.001	0.001	0.001	0.001	0.001	0.001

**Table 3:** Comparison of lymphocytes between newly diagnosed, relapsed, and refractory patients (*x̅* ± *s*, cells/*μ*L).

Group	*n*	CD3+	CD3+CD4+	CD3+CD8+	CD4+/CD8+	CD19+	CD16+CD56+	ALC (×109/L)
Newly diagnosed	48	603.90 ± 109.48	426.39 ± 24.82	687.45 ± 31.53	0.91 ± 0.39	365.17 ± 41.23	221.48 ± 24.98	3.97 ± 0.92
Relapse refractory	28	916.16 ± 126.88	587.59 ± 33.05	691.55 ± 34.85	1.31 ± 0.58	299.88 ± 32.05	287.69 ± 29.87	3.43 ± 0.65
*T*	—	11.307	24.121	0.526	3.592	7.199	10.363	2.730
*P* value	—	0.001	0.001	0.601	0.001	0.001	0.001	0.008

**Table 4:** Comparison of lymphocytes between newly diagnosed, relapsed, and refractory patients (*x̅* ± *s*, cells/*μ*L).

Group	*N*	CD3+	CD3+ CD4+	CD3+ CD8+	CD4+/CD8+	CD19+	CD16+ CD56+	ALC (×109/L)
Mild	41	836.86 ± 121.76	543.16 ± 39.88	648.33 ± 29.57	1.28 ± 0.71	309.61 ± 33.31	271.49 ± 30.88	3.41 ± 0.58
Severe	35	717.61 ± 109.01	418.56 ± 24.40	736.56 ± 36.48	0.80 ± 0.17	388.46 ± 43.15	215.86 ± 21.98	4.19 ± 1.10
*T*	—	4.464	16.083	11.644	3.902	8.982	8.902	3.946
*P*	—	0.001	0.001	0.001	0.001	0.001	0.001	0.001

**Table 5:** Diagnosis of absolute lymphocyte count in peripheral blood.

Group		Platelets combined with bone marrow examination	
		Positive (*n* = 76)	Negative (*n* = 80)
Absolute lymphocyte count	Positive	71	8
	Negative	5	72

**Table 6:** Diagnostic value of absolute peripheral blood lymphocyte count in primary immune thrombocytopenia.

Group	Sensitivity	Specificity	Positive prediction	Negative prediction
Absolute lymphocyte count	93.42% (71/76)	90.00% (72/80)	89.87% (71/79)	93.51% (72/77)

## Data Availability

The datasets used and analyzed during the current study are available from the corresponding author on reasonable request.
